The article "Optimized Tree Strategy with Principal Component Analysis Using Feature Selection-Based Classification for Newborn Infant's Jaundice Symptoms" was published in 2021. Journal: J Healthc Eng.

# Optimized Tree Strategy with Principal Component Analysis Using Feature Selection-Based Classification for Newborn Infant's Jaundice Symptoms

**DOI:** 10.1155/2021/9806011

**Published:** 2021-11-23

**Authors:** Debabrata Samanta, M. P. Karthikeyan, Marimuthu Karuppiah, Dalima Parwani, Manish Maheshwari, Piyush Kumar Shukla, Stephen Jeswinde Nuagah

**Affiliations:** ^1^Department of Computer Science, CHRIST Deemed to be University, Bangalore, India; ^2^Department of Computer Science, PPG College of Arts and Science, Coimbatore, India; ^3^Department of Computer Science and Engineering, SRM Institute of Science and Technology, Delhi-NCR Campus, Ghaziabad 201204, Uttar Pradesh, India; ^4^Sant Hirdaram Girls College Bhopal, Bhopal, Madhya Pradesh, India; ^5^Department of Computer Application, MCNUJC, Bhopal, Madhya Pradesh, India; ^6^Computer Science & Engineering Department, University Institute of Technology Rajiv Gandhi Proudyogiki Vishwavidyalaya (Technological University of Madhya Pradesh), Bhopal 462033, India; ^7^Department of Electrical Engineering, Tamale Technical University, Tamale, Ghana

## Abstract

One of the most important and difficult research fields is newborn jaundice grading. The mitotic count is an important component in determining the severity of newborn jaundice. The use of principal component analysis (PCA) feature selection and an optimal tree strategy classifier to produce automatic mitotic detection in histopathology images and grading is given. This study makes use of real-time and benchmark datasets, as well as specific approaches for detecting jaundice in newborn newborns. According to research, the quality of the feature may have a negative impact on categorization performance. Additionally, compressing the classification method for exclusive main properties can result in a classification performance bottleneck. As a result, identifying appropriate characteristics for training the classifier is required. By combining a feature selection method with a classification model, this is possible. The major outcomes of this study revealed that image processing techniques are critical for predicting neonatal hyperbilirubinemia. Image processing is a method of translating analogue images to digital formats and manipulating them. The primary goal of medical image processing is to collect information useful for disease detection, diagnosis, monitoring, and therapy. Image datasets can be used to validate the performance of newborn jaundice detection. When compared to conventional approaches, it offers results that are accurate, quick, and time efficient. Accuracy, sensitivity, and specificity, which are common performance indicators, were also predictive.

The article "Optimized Tree Strategy with Principal Component Analysis Using Feature Selection-Based Classification for Newborn Infant's Jaundice Symptoms" was published in 2021. Journal: J Healthc Eng.

## 1. Introduction

The idiom data mining can manage a massive volume of information, and the analytical skill overcomes the limitations in the existing data processing technologies. The frequent and expanding use of sensors, Internet, and heavy machines in a flying ratio has accelerated data on today's digital world. In big data analytics, data mining classification is seen as a vital and difficult topic to solve. Big data classification is the process of classifying data based on issues and challenges created by significant data controllers [1]. This primary reason for infant jaundice is an increase in the level of bilirubin. As the hemoglobin of red blood cells (RBC) in the womb is different than the hemoglobin after birth, the rate at which the new RBC produced is faster [2].

Furthermore, the infants' underdeveloped liver increases bilirubin level as fast as possible, and results in the hyperbilirubinemia are proposed [3]. In some instances, bilirubin's presence results in the following disorders: liver disease, viral infections, deficiency in enzymes, abnormality in RBC, hypothyroidism, and liver inflammation [4].

In [5], a BiliCam-based jaundice detection system is proposed for estimating newborn jaundice. The suggested system exploited the smartphone with the paper-based color calibration card for monitoring the jaundice in infants. An example of the projected BiliCam-based jaundice identification technique is represented in [6]. From this explanation, it is analyzed that the BiliCam exploits the built-in camera for photographing the newborn. After analyzing the data, the system uploads only the relevant portions in the image to the server. The server then detects the bilirubin levels by examining the skin of the newborn. Finally, the detection results are reported to the user for performing the necessary actions [7].

Detection of infant jaundice detection by detecting bilirubin concentration is based on two techniques, such as the invasive technique and noninvasive technique. In the invasive procedure, the physical examination is carried out to catch the swellings in the liver, legs, and ankles; then, based on the urine test results, the bilirubin concentration level is estimated. Whereas, in the noninvasive technique, the level of bilirubin is estimated using a transcutaneous bilirubin meter. This technique directs the light onto the neonate's skin and estimates the intensity of the wavelength returned. The transcutaneous bilirubin meter analyzes the reflected optical signal spectrum and then converts them into electrical signals using a photocell. The microprocessor's electrical signals represent the value of the generated serum bilirubin results conveyed by [7].

The article "Optimized Tree Strategy with Principal Component Analysis Using Feature Selection-Based Classification for Newborn Infant's Jaundice Symptoms" was published in 2021. Journal: J Healthc Eng.

When the bilirubin's value is within 6 mg/dl and 9 mg/dl, treating the jaundice will be more comfortable; else, it results in irreversible brain damage in the infants. Thus, detecting the jaundice in the early stages is mandatory. Generally, the infants are affected by the jaundice after discharging from the hospitals; hence, the parents perform the initial investigation for the presence of jaundice through visual assessment. As only the visual examination cannot determine the exact level of jaundice, an efficient system for detecting jaundice is essential [8]. In infant jaundice classification, the estimation of the bilirubin level using invasive techniques is considered a painful method because the blood samples are collected from the venipuncture. In this collection procedure, the small amount of blood that comes through the needle is maintained in the test tube [9, 10]. The critical drawbacks of invasive techniques are the introduction of additional infection risks due to venipuncture, underestimate or overestimate chances caused by the initial visual test, increased cost, lower efficiency for the hospitals, and increased time for obtaining the results. Thus, to address these issues, an efficient noninvasive technique is mandatory.  Figure 1 shows the general classification architecture for infant jaundice detection.

The BiliCam is an optimal noninvasive solution because it does not require any additional hardware [11]. The motivation behind the suggested research work is described in Section 3. Mitosis detection is a critical characteristic in detecting the extent of jaundice advancement as a result of these difficulties. For pathologists, recognising differences in nuclei and mitotic counties is difficult because to the following two factors: pathologists would create a large number of histopathological pictures since mitotic nuclei have the same size and shape as nonmitotic nuclei.

The technical difficulties faced during the implementation of the proposed method are complexity in collecting the dataset that contains jaundice-affected infants and normal infants and higher time consumption for the execution of the principle component analysis (PCA) in the research work [11]. This research's objectives include newborn jaundice detection by using the PCA-based time slot scheduling algorithm to provide better classification accuracy. The proposed research considers the problem of newborn infants' jaundice monitoring and detection using medical image processing. Then, the main contributions of the study are as follows. The key findings of this study showed that techniques of image processing are important for neonatal hyperbilirubinemia prediction. The main goal of this research is to acquire information related to illness identification, diagnosis, monitoring, and treatment. The standard performance measurements and comparative study with existing methods for output of the newborn jaundice detection using image datasets also demonstrated in this research work [12].

The article "Optimized Tree Strategy with Principal Component Analysis Using Feature Selection-Based Classification for Newborn Infant's Jaundice Symptoms" was published in 2021. Journal: J Healthc Eng.

The remainder of this study is represented as follows.  Section 2 provides the previous bilirubin detection for jaundice and its related work. Section 3 projects our system design.  Section 4 shows our experimental methodology. Finally, we conclude the work with future plan of research.

## 2. Related Works

In the medical field, the following study addresses jaundice image-based machine learning classification approaches. Image processing-based health outweighs structures make a significant contribution to improving clinical statistics structures through automation of patient event control and real-time medical record transmission. The fundamental thinking about the proposed rule is imitating higher and environment-friendly health capabilities in imitating the sufferers via imposing a networked information astronaut [13, 14]. The experts then documents that may want to fulfill this record concerning this record and yet supply a fast and efficient solution. The final mannequin will be properly outfitted with the applications where the physician executes a look at his patient from somewhere and any time explained. In the emergency scenario, the researchers imitated the ship's fortune letters. However, information obtained after consulting with a physician, such as the patient's current reputation and extensive clinical data, can be pondered over as well [15]. The proposed model can also be implemented as a mobile app, making it more accessible and convenient to access from anywhere on the planet. Furthermore, the system saves the child's customized measurements to an image-based fact shop in real-time. Preliminary checks regarding community overall performance on the jaundice software graph resulted in an average latency concerning 1.7 s and then rule arrival about 99.96%, therefore validating its usability. The jaundice classification based on prehepatic, hepatic, and posthepatic levels are explained in this section. The three-layer detection of the based group is overproduction, decreased conjugation, and decreased excretion (inter or extraobstruction). The bilirubin is calculated in chemical-based molecular chemical activity. Bilirubin is a tetrapyrrolic compound formed when the protoporphyrin ring breaks down (hemo). This structure has several isoforms, with bilirubin IX being the most important catabolite in vivo (near 99 percent). Other isoforms, such as II and XIII, are found in a much lower proportion in the bloodstream, despite the fact that the National Institute of Standards and Technology (NIST) reference material for bilirubin SRM 916 is no longer available, and other commercial preparations contain significant amounts of these two isoforms [15]. Still, chemical bilirubin detection consumed a long time detecting infant jaundice for a day or week data [7].  Figure 2 shows the hepatic-level-based bilirubin detection process.

The article "Optimized Tree Strategy with Principal Component Analysis Using Feature Selection-Based Classification for Newborn Infant's Jaundice Symptoms" was published in 2021. Journal: J Healthc Eng.

Figure 3 shows the working model that describes a chemical bond for under-five baby care proposed by [16]. A test experiment involves chemical monitoring and maintenance so well, so telemetry on sensor metering readings in imitation of a bird infrastructure has been raised or tested. Connectivity in a chemical enabled sensor/actuator node and a cellular application through a planet software has been proven and then examined within a variety of look at eventualities protected in the country and intercontinental areas as nicely as much a vehicular environment. The preliminary takes a look at protecting an odd node solely with sensors because of ambient conditions. In the subsequent phase, the sensors are because growth monitoring or essential symptoms pleasure stand chronic, described in quantity two proposed in [17]. Predictive modelling can play a vital role in analyzing large sets of population health information to identify the risks of a disease, allowing clinicians to avoid unnecessary therapies that may shorten a patient's life expectancy or have no effect at all. Malformation, damage, and disease are not the only causes of defects. The severity of the harm may be the result of jaundice abnormalities, but lobes have not been affected [16].  Figure 4 shows the infant jaundice detection using chemical-based RBC and cytochrome and unconjugated bilirubin. A total of 24 newborn patient datasets were supplied for the study, including both ictal and interictal data. Six-channel and 32-channel sets can be subdivided from these 24 sets. The standard worldwide 10–20 method was utilised to determine the placements of the surface electrodes. The first dataset was a sample of a single severe seizure (possibly atonic-clonic). The second set of data was an illustration of a complicated partial attack proposed by [18].

A widespread seizure occurred few minutes later in one hemisphere of the brain. At hertz, each of these datasets were sampled. The thought on that task got here by reducing the jaundice of patient in conformity with go-to per health practitioner on each epoch that necessity according to take a look at his pressure, bravery beat rate, and heat. With the help of that concept, both patients' time and then physicians are protected. Yet, medical doctors execute additionally assisting among fortune state of affairs as much as possible, explaining in [19]. The proposed solution to the problem is to assign good yet efficient medical capabilities to patients by connecting and gathering data records via health reputation monitors such as patient's morale rate, blood pressure, and ECG or to send a fortune warning in accordance with the patient's medical doctor's current reputation or complete scientific ID in [20].

The article "Optimized Tree Strategy with Principal Component Analysis Using Feature Selection-Based Classification for Newborn Infant's Jaundice Symptoms" was published in 2021. Journal: J Healthc Eng.

It would also stand profitable in imitation of examining a centralized system, the place every smart under-five medical institution booth inside a district and then vicinity transfer according to a chemical machine or its data facts store, which introduces extra hops of the transmission paths, including a distributed provision where every booth is directly related in imitation of the planet that has its records store, used to be the law among the preliminary study. The effect regarding the expansion on the provision performance choice afterward keeps in contrast with the impact. The preliminary studies have been proposed regarding the expansion on the provision performance [21]. The CT scan takes 20 minutes. After that, diagnoses started for patients and children. CT scans can help to cast off someone's sordid conditions or illnesses to that amount that bears symptoms comparable to CP. Finally, a CT scan displayed equally in imitation of an X-ray, yet parameter jaundice images about whole exclusive angles by allowing because of a precise analysis of several organs or tissues [22]. The listed existing approaches are consuming more prediction time, and there is lack of accuracy; it will lack the treatment that may cause the newborn baby death; this motive following the proposed computer-based instant result generates without delay.

## 3. System Design

The suggested jaundice detection system uses the images of the newborn babies for the skin detection module. This module converts the image in the RGB format to the grayscale format. As the skin detection module's output images are prone to salt and pepper noises, the hybrid median filter is deployed for removing the noises. The color and the pattern features are elaborated using the color models and the GLCM method from the filtered images. In the initial phase, the PCA combination with the optimized tree technique is proposed for the redundant feature elimination and complexity reduction. The proposed system depends on four major stages: feature extraction, classification, histopathological preprocessing, and jaundice color segmentation. The proposed system is designed based on the following main contributions. The proposed research considers the problem of newborn infants' jaundice monitoring and detection using medical image processing.

The article "Optimized Tree Strategy with Principal Component Analysis Using Feature Selection-Based Classification for Newborn Infant's Jaundice Symptoms" was published in 2021. Journal: J Healthc Eng.

The ability to accommodate different feature selection criteria and locate certain tiny subsets of features that work well for a specific inductive learning method of interest to create the classifier is one of this analysis's strengths.

The main goal is to successfully use data from various feature selection methods to select better feature subsets with smaller sizes and better classification performance than existing methods.

### 3.1. Skin Detection

The performance of skin detection depends on the color space, model, and classification method. Choosing a color space is an essential criterion in skin detection, a critical task for real-time applications. The disparate color spaces such as the RGB model, YUV, or YCbCr are used in this research work. The RGB is a typical choice to represent the color image, which is extensively used in various systems. YUV or YCbCr color spaces are commonly used for real-time skin detection, and the transformation between YUV and RGB is linear. The luma component of the color is represented by Y. The color's brightness is measured in luma. This refers to the color's light intensity. This component is more sensitive to the human sight. Cb and Cr are the blue and red components of the chroma component, respectively. “Cb is the blue component in relation to the green component, and Cr is the red component in relation to the green component,” says the definition. The human eye is less sensitive to these components. Dataset collected newborn infant child for both jaundice and nonjaundice presented image.

In this research work, the input infant image is converted from RGB to grayscale and grayscale to binary. From the altered images, the region of interest (ROI) crops the necessary portions from the skin area. The cropped part was subjected to the hybrid median filter for removing the noise.  Figure 5 shows the proposed infant newborn jaundice prediction architecture diagram.

The fundamental goal of developing a jaundice classification technique is to construct mathematical demonstrations and minimise input data, so that the input signal can be appropriately classified. In a way, these mathematical representations of movement constitute a mapping of a multidimensional gap with different input signals into a smaller area. “Feature extraction” is the term for this dimensional reduction. Finally, just the most significant data from the original signal should be kept in the extracted feature set.  Figure 4 shows the proposed newborn infant jaundice detection block diagram.

The article "Optimized Tree Strategy with Principal Component Analysis Using Feature Selection-Based Classification for Newborn Infant's Jaundice Symptoms" was published in 2021. Journal: J Healthc Eng.

### 3.2. Preprocessing

Median: all the grey level values are arranged in ascending order, and then, the midpoint value of the grey level is called the median of the candidate region.

(1) $$\begin{array}{c} \text{SD}=\sqrt{\frac{1}{N-1}\sum_{i=1}^{N}{\left(x_{i}-\bar{x}\right)}^{2}}. \end{array}$$

The noises present in the image degrade the detection system's performance, so it must be denoised before processing the images. Here, the hybrid median filtering algorithm is employed to denoise the given input baby image.

### 3.3. Segmentation

The jaundice picture is extracted using the bounding box (a patch of 120 × 120 pixels). The accuracy of segmentation, preprocessing of histopathology images, and the time it takes for segmentation to become predictable are all affected by picture capture quality. Nuclei from these patches are subsequently segmented using an expectation-maximization technique (EM).

(2) $$\begin{array}{c} P\left(\omega c|f\left(p\right)\right)=\frac{\mathrm{PcN}\left(f\left(p\right)|\mu c,\Sigma c\right)}{\sum_{i=1}^{C}\mathrm{PiN}\left(f\left(p\right)|\mu c,\Sigma i\right)}. \end{array}$$

### 3.4. Feature Extraction

Three methods categorize histopathological images. The first way is newborn jaundice segmentation, which denotes cellular alterations, the second technique is based on textural properties, and the third method is based on color density differences. Feature elaboration is the process of transforming the contents of the image into multiple content features. The suggested jaundice detection system extracts two types of features such as texture and shape features and intensity features.

The GLCM feature extraction algorithm is proposed for extracting the texture and shape features and intensity features. The suggested GLCM feature extraction algorithm identifies the specific characteristics of newborn infant jaundice detection. Extraction of image features is shown in Figure 6.

## 4. Proposed Methodology

In this section, we will discuss methodology for the PCA feature selection mechanism to classify newborn infant's jaundice with an optimized tree strategy. We consider newborn baby images as input data. The baby (child) image recognizes jaundice or not (Algorithm 1).

## 5. Result Analysis and Discussion

### 5.1. Results

Matlab 2013a is used to implement the proposed methodology on an Intel(R) Core (TM) i5-2410M CPU 2.30 GHz with 16 GB RAM. The performance of the researcher suggested principal component analysis-based optimal tree strategy (PCATOS) is evaluated using infant jaundice detection as a case study since it has an impact on lifetime motion incapacity. The facts about jaundice are gathered in a variety of methods from a variety of unsorted sources. The testing data provided by the Kaggle dataset was used for this initial testing. The data from the neonatal jaundice prediction project are used in all following investigations. This was done since it was easier to assess the system's accuracy by looking at multiple seizure cases from the same patient, especially a youngster. The second phase experiment aimed to find a preictal state duration that best exposed the qualities that lead to the condition of jaundice impact.

The article "Optimized Tree Strategy with Principal Component Analysis Using Feature Selection-Based Classification for Newborn Infant's Jaundice Symptoms" was published in 2021. Journal: J Healthc Eng.

The preprocessing step seeks to improve the image collection by reducing irregular disturbances and evaluating some significant picture patterns for further processing. The training and testing data in this experiment are unconnected and from various newborn jaundice datasets, but they are all recorded and used to discover the best feature sets that maximise prediction accuracy. These tests demonstrate the relative strength of each categorization algorithm and approximate the behaviour of state transitions.

Image of jaundice: as the pixel of the image starts to the end pixel, a different set of data's colors is prominent, and preprocessing activity is often simple to notice visually in an input image appearance. This provided as a simple sign of how the planned prediction system worked. Because there is no gold standard for distinguishing between individual states in pattern recognition, an initial guess of *t* states was defined in jaundice or not. The proposed system result obtained matrix results are given in Table 1 and Figure 5.

Using the knowledge gathered from previous tests, a balance of all the algorithms characteristics, as well as other parameters, a prediction model capable of identifying the jaundice state was developed as given in Table 1 that described confusion matrix values. The total amounts classified in two actual and predicted jaundice values are separated as usual and jaundice. Based on Table 1 values, the following performance evaluations are measured and the proposed system is compared to the logistic regression and K-nearest neighbor approaches.

### 5.2. Discussion

The performance measure for PCATOS is given in Table 1. In this proposed analysis, the efficiency percentage is increased. In this proposed work, the accuracy and classification rate level increased compared to the previous approach. The outcomes of this experiment demonstrated the utility of the state decision PCA for making state transitions and improving categorization.

Table 2 provides the comparative analysis of the accuracy of the existing logistic regression, logistic regression, and proposed principal component analysis-based optimized tree strategy.  Figure 7 shows the comparison of precision of the current technique with the proposed principal component analysis-based optimized tree strategy (PCAOTS). The figure shows that the accuracy of the proposed PCAOTS is higher than the existing techniques.

The article "Optimized Tree Strategy with Principal Component Analysis Using Feature Selection-Based Classification for Newborn Infant's Jaundice Symptoms" was published in 2021. Journal: J Healthc Eng.

Table 3 provides the comparative analysis of sensitivity for the principal component analysis-based optimized tree strategy (PCAOTS), logistic regression and K-NN-based FS method. The sensitivity of the existing PCAOTS is 96.2%, K-NN-established FS method is 92.4%, and logistic regression is only 64.3%.  Figure 8 shows the sensitivity analysis plot for PCAOTS, K-NN-based FS method, and logistic regression. From Figure 8, it is observed that the proposed PCA-based optimized tree strategy has a high sensitivity value than the existing process.

Table 4 and Figure 9 show the comparison results of the existing logistic regression, K-NN-based FS method, and PCA-based optimized tree strategy. The specificity of the existing logistic regression is 81%, K-NN found the FS method is 95%, and the PCA-based optimized tree strategy is 98%. In the proposed way, high specificity is attained by implementing the PCA-based FS method approach.

The research has been thoroughly tested, and positive results have been obtained. After confirming the findings, it was discovered that designed research may be used to diagnose jaundice in real-time with no errors. As a result of seeing the results, appropriate steps are performed to avoid the child's health condition from deteriorating further. The system is capable of providing real-time solutions to difficulties, and the perfect achievement is achieved without delay.

## 6. Conclusion and Future Works

In this research study, detecting the variations of colors in a particular histopathological image area is essential in predicting newborn jaundice's progression. Segmentation of the jaundice image is a great challenge due to shape, varying size, and nonhomogenous pixel intensity present in the picture. A study of the best feature sets for accuracy was performed. Finally, an emulator was used to compare three algorithm outcomes in a real-time setting using mat abide with a single channel to the frontal lobe of the face. Several kinds of research stated about newborn jaundice diseases detection, but lack in accurately extracting the newborn jaundice. This proposed method, automatic newborn jaundice detection in histopathology images and grading using the PCA feature selection mechanism to classification for newborn infant's jaundice with an optimized tree strategy yields an accuracy 95%, specificity 96%, and sensitivity 98%. The proposed system of principal component analysis-based optimized tree strategy attains better accuracy in terms of efficiency and time duration. The following features need to consider further implementation for jaundice detection: feature selection methods such as rough set theory incorporating machine learning approaches need more research. Lot of work is to be done to the soft set-based classifiers for the high dimensional database.

The article "Optimized Tree Strategy with Principal Component Analysis Using Feature Selection-Based Classification for Newborn Infant's Jaundice Symptoms" was published in 2021. Journal: J Healthc Eng.

## Figures and Tables

**Figure 1:** Steps involved in jaundice detection image processing.

**Figure 2:** Bilirubin detection process hepatic level based.

**Figure 3:** Hyperbilirubinemia neonatal jaundice detection process.

**Figure 4:** Proposed newborn infant jaundice detection block diagram.

**Figure 5:** Proposed infant newborn jaundice prediction architecture diagram.

**Figure 6:** Extraction of image features.

**Figure 7:** Accuracy comparison graph for the newborn jaundice dataset.

**Figure 8:** Sensitivity comparisons graph for the newborn jaundice dataset.

**Figure 9:** Specificity comparison graph for the newborn jaundice dataset.

**Algorithm 1:** PCA-based optimized tree strategy.

**Table 1:** Confusion matrix.

Confusion matrix		Predicted	
		Normal	Jaundice
Actual	Normal	63	4
	Jaundice	3	72

**Table 2:** Accuracy comparison for the newborn jaundice dataset.

Methods	Accuracy (%)
Logistic regression (LR)	92.5
K-NN	94.2
PCAOTS	95.5

**Table 3:** Sensitivity comparison for the newborn jaundice dataset.

Methods	Sensitivity (%)
Logistic regression	64.3
K-NN	92.4
PCAOTS	96.2

**Table 4:** Specificity comparison for the newborn jaundice dataset.

Methods	Specificity (%)
Logistic regression	81
K-NN	95
PCAOTS	98

## Data Availability

The newborn patient image data used to support the findings of this study are available from the corresponding author upon request.
